RETRACTED

# Computational Study on the Inhibitory Effect of Natural Compounds against the SARS-CoV-2 Proteins

**DOI:** 10.1155/2022/8635054

**Published:** 2022-03-25

**Authors:** John Marshal Jayaraj, Muralidharan Jothimani, Chella Perumal Palanisamy, Olli T. Pentikäinen, Mehboobali Pannipara, Abdullah G. Al-Sehemi, Karthikeyan Muthusamy, Krishnasamy Gopinath

**Affiliations:** ^1^Pharmacogenomics and CADD Lab, Department of Bioinformatics, Alagappa University, Karaikudi, Tamil Nadu, India; ^2^State Key Laboratory of Biobased Materials and Green Paper Making, School of Food Science and Engineering, Qilu University of Technology, Shandong Academy of Sciences, Jinan, Shandong, China; ^3^Faculty of Medicine, Integrative Physiology and Pharmacology, Institute of Biomedicine, University of Turku, Turku, Finland; ^4^Research Centre for Advanced Materials Science, King Khalid University, Abha 61413, Saudi Arabia; ^5^Department of Chemistry, King Khalid University, Abha 61413, Saudi Arabia

## Abstract

COVID-19 is more virulent and challenging to human life. In India, the Ministry of AYUSH recommended some strategies through Siddha, homeopathy, and other methods to effectively manage COVID-19 (Guidelines for AYUSH Clinical Studies in COVID-19, 2020). *Kabasura Kudineer* and homeopathy medicines are in use for the prevention and treatment of COVID-19 infection; however, the mechanism of action is less explored. This study aims to understand the antagonist activity of natural compounds found in Kabasura Kudineer and homeopathy medicines against the SARS-CoV-2 using computational methods. Potential compounds were screened against NSP-12, NSP-13, NSP-14, NSP-15, main protease, and spike proteins. Structure-based virtual screening results shows that, out of 14,682 Kabasura Kudineer compounds, the 250395, 129677029, 44259583, 44259584, and 88583189 compounds and, out of 3,112 homeopathy compounds, the 3802778, 320361, 5315832, 14590080, and 74029795 compounds have good scoring function against the SARS-CoV-2 structural and nonstructural proteins. As a result of docking, homeopathy compounds have a docking score ranging from −5.636 to 13.631 kcal/mol, while Kabasura Kudineer compounds have a docking score varying from −8.290 to −13.759 kcal/mol. It has been found that the selected compounds bind well to the active site of SARS-CoV-2 proteins and form hydrogen bonds. The molecular dynamics simulation study shows that the selected compounds have maintained stable conformation in the simulation period and interact with the target. This study supports the antagonist activity of natural compounds from Kabasura Kudineer and homeopathy against SARS-CoV-2's structural and nonstructural proteins.

RETRACTED

## 1. Introduction

The deadly pathogen causing novel coronavirus disease 2019 (COVID-19) became more virulent and resistant to the medicine and vaccines; still, a more effective management system and medicines might be required to effectively manage COVID-19 [1]. The pathogenic coronaviruses that affect humans, that is, SARS-CoV-1, the Middle Eastern respiratory syndrome coronavirus (MERS-CoV), and recent SARS-CoV-2 all belong to the beta coronaviruses group [2]. SARS-CoV-2 is an enveloped virus with a positive sense and single-stranded RNA genome [3], which emerged in bats, but it may have been augmented in an intermediary host and used an angiotensin-converting enzyme 2 (ACE2) from bats, civet cats, swine, cats, ferrets, nonhuman primates (NHPs), and humans as a receptor [4, 5]. The spike protein's receptor-binding domain (RBD) is the most erratic component of the coronavirus genome. The six amino acids present in them play a vital role in binding to ACE2 receptors; they are Y442, L472, N479, D480, T487, and Y4911 residues in SARS-CoV-2 and L455, F486, Q493, S494, N501, and Y505 residues in SARS-CoV-2. Furthermore, the SARS-CoV-2 seems to have an RBD that possesses a good binding affinity to ACE-2 from humans, ferrets, cats, and other species. The delta plus variant has an additional mutation on the coronavirus spike called K417N, which was first discovered in South Africa and Brazil, respectively. (Beta was linked to increased hospitalization and deaths during South Africa's first wave of infections. Gamma was estimated to be highly transmissible.) Mutations occur over time, and the virus adapts to new viral properties to enhance its spread. Among these viral variants, alpha (*α*), beta (*β*), gamma (*γ*), delta (*δ*), and omicron are transmitting in more significant numbers and causing a reduction in vaccine effectiveness. The recently identified variant called omicron was found in South Africa in November 2021. It consisted of 32 mutations, whereas alpha, beta, and gamma only contained 13, 10, and 11 mutations for each. Only 15 mutations were found in the receptor-binding domain (RBD) of omicron out of 32 types. The omicron viral spread is very high on a global scale and causes many death cases. Overall, the SARS-CoV-2 pandemic is continuing, so we need to identify the molecular mechanism of disease as well as a potent medication for this COVID-19 as soon as possible.

Siddha medicine is one of the conventional medicines, which was habitually used in Tamil Nadu, South India. As per the report stated by the Siddha medicine, the disease occurs due to variation of *tridoshas*, namely, *vatha*, *pitha*, and *kapha*. In an individual human being, the three different biological mechanisms of vatha, pitha, and kapha was cured by using an herb, metals, and minerals [6, 7]. The prevention and treatment of viral infections based on the accessibility of antiviral drugs are very few, and it is quite a tough challenge to prevent viral replication, but the Siddha herbal components have shown possible effects against influenza, dengue, chikungunya, tuberculosis, and so on [8, 9]. Overall, 32 internal medicines and 2 Siddha medicines such as *Kabasura Kudineer* and *Nilavembu Kudineer* are suggested by the Government of India against the viral infections of COVID-19, swine flu, dengue, and chikungunya [10]. Kabasura Kudineer is a polyherbal Siddha formulation with 15 ingredients and is prescribed widely for its effective administration against respiratory infections such as cold, cough, breathing difficulty, and flu [11]. COVID-19 infections commonly cause multipathogenic complications and affect the vital organ system of humans. The polyherbal compounds of the Kabasura Kudineer control the COVID-19 infections effectively and protect the other organ system; it may play on multiple target proteins. Samuel Hahnemann demonstrated homeopathy in 1976. He treated himself with some amount of cinchona tree bark that contains the drug quinine that cures malaria [7]. So we screened a huge set of Kabasura Kudineer and homeopathy compounds that possess antiviral activity against the novel corona virus in a very short era.

RETRACTED

A drug design approach can lead to more time-consuming and less cost-effective drug molecules against SARS-CoV-2. The main objective of the study was to identify compounds that could inhibit the SARS-CoV-2 proteins using Kabasura Kudineer and homeopathy compounds. Here, we used various computational approaches to identify a potent inhibitor against SARS-CoV-2. Initially, we retrieved the SARS-CoV-2 protein structure from the Protein Data Bank (PDB) and the structure of the natural compounds from the PubChem database. We then applied a structure-based virtual screening (SBVS) approach to each compound and protein. We selected the best compounds for DFT analysis from SBVS results. The electrostatic potential and orbital transferring abilities of the best-taken compounds were investigated through DFT analysis. The molecular dynamics study governed the molecular stability, conformational changes, and interaction patterns.

## 2. Materials and Methods

All the computational and molecular dynamics studies were conceded by the centos v7.0 Linux platform with Intel®core™ i7-4470 CPU @ 3.40 GHz processor alongside the installed software package (Schrödinger, LLC, New York, 2018-4). The several SARS-CoV-2 structural (spike and membrane protein) and nonstructural proteins (main protease, NSP-12, NSP-13, NSP-14, and NSP-15) were preferred as targets to perform docking analysis against SARS-CoV-2 with different compounds by using Maestro (Schrödinger 2018-4) [12, 13].

RETRACTED

### 2.1. Data Set

The targeted proteins structures were taken from the Protein Data Bank (RCSB-PDB). The protein structures are crucial for mounting the drug molecule against SARS-CoV-2. The targeted proteins structures are main protease (PDB ID: 6LU7) [14], spike protein (PDB ID: 7BZ5) [15], NSP-12 (PDB ID: 6XQB) [16], NSP-13 (PDB ID: 5WWP) [17], NSP-14 (PDB ID: 5C8S) [18], and NSP-15 (PDB ID: 6X4I) [13, 19, 20]. The SARS-CoV-2 membrane protein was not available in the Protein Data Bank. The membrane protein was modeled by the I-tasser server [21]. To intend the drug for rising SARS-CoV-2, we need a huge set of Kabasura Kudineer and the homeopathy compounds; these compounds were downloaded from the PubChem library database (https://pubchem.ncbi.nlm.nih.gov/).

### 2.2. Protein Structure Preparation and Active Site Generation

The X-ray crystal structures of SARS-CoV-2 main protease, spike protein, NSP-12, NSP-13, NSP-14, NSP-15, and membrane protein were prepared using Schrödinger 2018-4 server. The X-ray crystal structure was imported in the protein preparation wizard of Maestro (Schrödinger 2018-4). The crystal structure residues of the atoms were missing, and the protein side-chain and bond order varied. The protein missing atoms were added, and the water molecules were removed by Schrödinger 2018-4. Furthermore, the structures were optimized and minimized through the OPLS3 force field; the targeted protein does not contain a cocrystal ligand. So the site map was generated by the sitemap module of Schrödinger 2018-4. The top-scoring sites were chosen for a receptor-grid generation. The grid generation was performed with a default panel that set the inner box to 10 × 10 × 10 Ǻ by glide grid module of Schrödinger 2018-4, generated by an active site, and recognized the amino acid position in the protein. The grid file was used for virtual screening workflow to categorize a potential compound [22].

### 2.3. Ligand Preparation

The Kabasura Kudineer and homeopathy compounds were retrieved from the PubChem database (http://pubchem.ncbi.nlm.nih.gov/). Furthermore, the compounds were prepared by using LigPrep module of Schrödinger 2018-4. Overall, 1,000 conformers were generated in each compound in the preprocess (100-step) and postprocess (50) minimization steps, which were performed using the OPLS3 force field. This conformer was filtered by relative energy than a window of 10 kcal/mol, and the minimum atom deviation range is 1 Å. High energy conformers were removed; the ligands were prepared; and these conformers were generated [23].

RETRACTED

### 2.4. Virtual Screening Study

The SARS-CoV-2 targeted proteins and prepared compounds (Kabasura Kudineer and homeopathy) were used for structure-based virtual screening (SBVS) workflow. SBVS workflow was done using a Virtual Screening Workflow Suite, Maestro, Schrödinger 2018-4, using OPLS3 force field. Through Lipinski's rule of five and ADME calculations by QikProp, violation compounds were initially filtered through a collection of data sets. Furthermore, the compounds were screened by docking procedures such as high throughput virtual screening (HTVS), standard precision (SP), and extra precision (XP) mode screening methods in the virtual screening workflow of Maestro, Schrödinger 2018-4. The top hit compounds were selected by taking the glide score, glide energy, and hydrogen bond interactions [24].

### 2.5. Density-Functional Theory (DFT) Calculations

The density-functional theory (DFT) calculations were performed on the top hit compounds using the virtual screening procedure. We have studied the electronic molecular features, including frontier molecular orbitals (HOMO and LUMO) and electrostatic potential and density, using DFT calculations that might demonstrate the molecular electronic features. The DFT analysis was performed by the Jaguar module (Schrödinger, LLC, New York, 2018-4). In the DFT computation, Becke's three-parameter via Lee Yang Parr correlation functional (B3LYP) and basis set 6-31G*∗∗* was used to calculate the MESP, HOMO, and LUMO of the selected compounds. The highest occupied molecular orbital (HOMO) and the lowest unoccupied molecular orbital (LUMO) energy revealed the energy gap of ligand that was indicated as an electron transition energy, and it plays a significant role in analyzing the ligand stability and reactivity [25, 26]. The color-coded MESP surface indicates the positive and negative potential in blue and red colors. The reactivity range shows yellow, orange, and green colors.

### 2.6. Molecular Dynamic Simulation Study

Molecular dynamics simulation was performed in Desmond (Schrödinger, LLC, New York, USA; Desmond, Schrödinger, 2019). Desmond employed the neutral territory approach, commonly known as the midway method. This was accomplished with skillful use of a high level of computing parallelism. The SARS-CoV-2 structural and nonstructural proteins structural stability and flexibility were predicted using Desmond. The TIP3P force field was used to obtain energy minimization and optimization. Desmond was used to run a molecular dynamics (MD) simulation of SARS-CoV-2 structural and nonstructural proteins to test the stiffness of the protein and ligand combination. The docked protein-ligand complexes were solved using a system builder using the simple point energy (SPC), a water mode in an orthorhombic box. The crossing water molecules were removed. The system was counteracted with an appropriate amount of Na^+^/cl^−^ counter ions with a permanent salt concentration of 0.15 M depending on the system's full charge. To improve the stability, the primed system was agreed with the default relaxation procedure contained in the Desmond to run molecular dynamics simulations for 100 ns with a random condition in the number of atoms, pressure, and temperature (NPT) ensemble. Furthermore, the best inhibitors were taken for molecular dynamics (MD) simulation studies. The protein stability is examined by calculating the RMSD, RMSF, and interaction analysis [27–29].

RETRACTED

## 3. Results and Discussion

### 3.1. Virtual Screening Study

Virtual screening workflow was performed using Schrödinger suite from Kabasura Kudineer, homeopathy compounds against SARS-CoV-2 structural and nonstructural proteins. The SARS-CoV-2 structural and nonstructural proteins were the points of concern in transcription, translation, synthesis, virus replication, and infection. SARS-CoV-2 PLpro was liable for dividing the N-terminus of the replicase polyprotein to discharge NSP1, NSP2, and NSP3, which play a vital role in the virus replication. 3CLpro (chymotrypsin-like protease), also known as Nsp5, was robotically cleaved from polyprotein to generate enzymes and further divides Nsps downstream at 11 sites to free Nsp4 and Nsp6. Nsp12 is an RNA-dependent RNA polymerase (RdRp) that plays a role in virus replication and polymerization of viral RNA having a deep cavity as an active site. Nsp13 is a multifunctional helicase having a zinc-binding domain at the N terminus that can unwind RNA and DNA duplexes with 5′ to 3′ polarity. The Helicase activity is influenced by magnesium; Nsp14 has an exoribonuclease activity that acts in the 3′ to 5′ direction on both ssRNA and dsRNA; and an N7-guanine methyltransferase activity and Nsp15 is a uridylate-specific endoribonuclease that cleaves 2′-3′-cyclic phosphates 5′ to the cleaved bond. It is Mn2+-dependent and uridylate-specific. Since the study was mainly focused on the SARS-CoV-2 structural proteins such as membrane protein, spike protein (PDB ID: 7BZ5), and nonstructural proteins such as the main protease (PDB ID: 6LU7), Nsp12 (PDB ID: 6XQB), Nsp13 (PDB ID: 5WWP), Nsp14 (PDB ID: 5C8S), and Nsp15 (PDB ID: 6X4I) as potential target proteins for SARS-CoV-2. Therefore, these proteins were a significant target to develop inhibitors against SARS-CoV-2 [7].

RETRACTED

A total of 14,682 Kabasura Kudineer and 3,112 homeopathy compounds were obtained from the PubChem database. But all the compounds were filtered out depending on the Lipinski rule of five calculations. Still, the rule of five classifies the molecules that rely on the molecular weight ≤ 500, clogP ≤ 5, H-bond donor ≤ 5, and H-bond acceptor ≤ 1. The filtered compounds were utilizing a VSW. Overall, 192 Kabasura Kudineer and 515 homeopathy filtered compounds were screened with SARS-CoV-2 structural and nonstructural protein. Finally, the best five inhibiting compounds were determined based on the docking score. As a result, compared to other compounds, 250395, 129677029, 44259583, 44259584, and 88583189 (Kabasura Kudineer) and the 3802778, 320361, 5315832, 14590080, and 74029795 (homeopathy) compounds had a strong scoring function with SARS-CoV-2 structural and nonstructural protein. The top five homeopathy compounds docking score ranged from −13.631 to −5.636 kcal/mol, while the top five Kabasura Kudineer compounds docking score ranged from −13.791 to −7.273 kcal/mol.

### 3.2. Virtual Screening Study of SARS-CoV-2 Structural and Nonstructural Proteins with Homeopathy Compounds

A huge set of homeopathic compounds were docked with the structural and nonstructural proteins of SARS-CoV-2. As a result, when compared to other compounds, the homeopathic compounds 3802778, 320361, 5315832, 14590080, and 74029795 had an excellent scoring function with SARS-CoV-2 protein. The 14590080 compound has a high binding score (−13.631 kcal/mol) compared to the other four compounds (Table 1).

### 3.3. Binding Mode Analysis of Homeopathy Compounds

The binding modes of the best compounds were analyzed by the Glide XP module. The binding mode analysis of the best five compounds image was given in Figure 1.

#### 3.3.1. Binding Mode Analysis of the Compound 3802778

The 3802778 compound had a docking score of −7.929 kcal/mol and was bound with SARS-CoV-2 spike protein. The respective compound interacts with Arg355 and Asp428 residues. In Arg355, (H…OH) hydrogen interacted with the oxygen group, which distance is 2.04 Ǻ. The Asp428 (H…OH) hydrogen interacted with the oxygen group, which distance is 1.83 Ǻ, and same (H…OH) hydrogen residues interacted with the oxygen group, and the distance was noted as 1.69 Ǻ. The residues interactions play a major role in SARS-CoV-2 protein antagonist activity.

#### 3.3.2. Binding Mode Analysis of the Compound 3802778

The 3802778 compound had a docking score of −9.583 kcal/mol and was bound with SARS-CoV-2 Nsp14. The respective compound interacts with Lys93, Gly94, Ala71, Asn40, and Lys95 residues. In Lys93, (H…OH) hydrogen interacted with the oxygen group of 3802778 compound, and the distance was 2.00Ǻ, and the same residues having pi-pi interactions, this pi-pi interaction was strong for stable binding of a compound in the active site of SARS-CoV-2. In Gly94, (H…OH) hydrogen interacted with the oxygen, and the distance was 2.20 Ǻ. In Ala71, (H…OH) hydrogen interacted with the oxygen group, and the distance was 2.57 Ǻ, and in the same residues, (H…OH) hydrogen interacted with the oxygen group, and the distance was 1.84 Ǻ. In Asn40, (H…OH) hydrogen interacted with the oxygen group, and the distance was 1.86 Ǻ. In Lys95, (H…OH) hydrogen interacted with the oxygen group, and the distance was 1.96 Ǻ, and in the same residues, (H…OH) hydrogen interacted with the oxygen group, and the distance was 1.81 Ǻ. The residues interactions play a major role in SARS-CoV-2 protein antagonist activity.

RETRACTED

#### 3.3.3. Binding Mode Analysis of the Compound 320361

The compound 320361 had a docking score of –5.636 kcal/mol and was bound to SARS-CoV-2 Membrane protein. The respective compound interacted with Tyr61 residues. In Tyr61, the residues were formed with three hydrogen bond interactions with 320361 compounds. In Tyr61, (H…OH) hydrogen interacted with the oxygen, and the distance was noted as 2.01 Ǻ; (H…OH) hydrogen interacted with the oxygen group, and the distance was noted as 2.11 Ǻ; and (H…OH) hydrogen interacted with the oxygen group, and the distance was noted as 2.05 Ǻ. The residues interactions play a major role in SARS-CoV-2 protein antagonist activity.

#### 3.3.4. Binding Mode Analysis of the Compound 5315832

The 5315832 compound had a docking score of −7.672 kcal/mol and was bound with SARS-CoV-2 Nsp14. The respective compound interacts with Thr5, Asn40, Tyr96, Ala71, Lys95, and Gly94 residues. In Thr5, (H…OH) hydrogen interacted with the oxygen group of 5315832 compound, and the observed distance was 2.07 Ǻ; Tyr96 residues have pi-pi interactions, and these pi-pi interactions were strong for stable binding of the compound in the active site of SARS-CoV-2. In Asn40, (H…OH) hydrogen interacted with the oxygen, and the distance was 2.72 Ǻ. In Ala71, (H…OH) hydrogen interacted with the oxygen group with a distance of 2.58 Ǻ. In Lys95, (H…OH) hydrogen interacted with the oxygen group at a distance of 1.98 Ǻ, and in the same residues, (H…OH) hydrogen residues interacted with the oxygen group at a distance of 1.97 Ǻ. In Gly94, (H…OH) hydrogen interacted with the oxygen group with a distance of 2.25 Ǻ; the residues interactions play a major role in SARS-CoV-2 protein antagonist activity.

#### 3.3.5. Binding Mode Analysis of the Compound 14590080

The 14590080 compound had a docking score of −13.631 kcal/mol and found to bind with SARS-CoV-2 Nsp13. The respective compound interacts with Ser539, Ser535, Gln531, Thr530, and Asn516 residues. In Ser539, (H…OH) hydrogen interacted with the oxygen at a distance of 1.94 Ǻ. In Ser535, the residues formed three hydrogen bond interactions with 14590080 compound, and (H…OH) hydrogen interacted with the oxygen group at a distance of 1.89 Ǻ, In Thr701, (H…OH) hydrogen interacted with the oxygen at a distance of 1.92 Ǻ. In Thr701, (H…OH) hydrogen interacted with the oxygen at a distance 2.05 Ǻ. In Gln531, (H…OH) hydrogen interacted with the oxygen at a distance of 2.13 Ǻ. In Thr530, (H…OH) hydrogen interacted with the oxygen group, at a distance of 2.08 Ǻ, and in the same residues, (H…OH) hydrogen interacted with the oxygen group at a distance of 2.69 Ǻ. In Asn516, (H…OH) hydrogen interacted with the oxygen group at a distance of 2.03 Ǻ. The residues interactions play a major role in SARS-CoV-2 protein antagonist activity.

RETRACTED

#### 3.3.6. Binding Mode Analysis of the Compound 74029795

The 74029795 compound was having a docking score of –11.957, kcal/mol and was bound with SARS-CoV-2 Nsp13. The respective compound interacts with Ser539, Ser537, and Ser535 residues. In Ser539, (H…OH) hydrogen interacted with the oxygen group at a distance of 2.01 Ǻ. In Ser537, (H…OH) hydrogen interacted with the oxygen group at a distance of 1.90 Ǻ, and in the same residues, (H…OH) Hydrogen interacted with the oxygen group at a distance of 2.14 Ǻ. In Ser535, (H…OH) hydrogen interacted with the oxygen group at a distance of 1.80 Ǻ. The residues interactions play a major role in SARS-CoV-2 protein antagonist activity.

#### 3.3.7. Binding Mode Analysis of the Compound 74029795

The 74029795compound was having a docking score of −8.637 kcal/mol, and it was binding with SARS-CoV-2 main protease. The respective compound interacts with Gln189, Asn142, and Gly143 residues. In Gln189, the residues were formed by three hydrogen bond interactions with 74029795 compounds; (H…OH) hydrogen interacted with the oxygen at a distance of 2.02 Ǻ; (H…OH) hydrogen interacted with the oxygen group at a distance of 1.83 Ǻ; and (H…OH) hydrogen interacted with the oxygen group at a distance of 1.89 Ǻ. In Asn142, (H…OH) hydrogen interacted with the oxygen group at a distance of 1.91 Ǻ. In Gly143, (H…OH) hydrogen interacted with the oxygen group at a distance of 2.04 Ǻ. The residues interactions play a major role in SARS-CoV-2 protein antagonist activity.

#### 3.3.8. Binding Mode Analysis of the Compound 3802778

The 3802778 compound had a docking score of −10.902 kcal/mol and was bound with SARS-CoV-2 Nsp12. The respective compound interacts with Asn297, Ser274, Thr275, Lys71, Tyr279, Glu69, Ser198, and Gln202 residues. In Asn297, (H…OH) hydrogen interacted with the oxygen group of 3802778 compound at a distance of 2.15 Ǻ. In Ser274, (H…OH) hydrogen interacted with the oxygen at a distance of 2.26 Ǻ. In Thr275, (H…OH) hydrogen interacted with the oxygen group at a distance of 1.72 Ǻ. In Lys71, (H…OH) hydrogen interacted with the oxygen group at a distance of 2.15 Ǻ. In Tyr279 residues, (H…OH) hydrogen interacted with the oxygen group at a distance of 1.91 Ǻ. In Glu69, (H…OH) hydrogen interacted with the oxygen group at a distance of 2.16 Ǻ. In Ser198, (H…OH) hydrogen interacted with the oxygen group at a distance of 1.94 Ǻ, and in Gln202, (H…OH^−^) hydrogen interacted with the oxygen group at a distance of 2.05 Ǻ. The residues interactions play a major role in SARS-CoV-2 protein antagonist activity.

RETRACTED

#### 3.3.9. Binding Mode Analysis of the Compound 320361

The 320361compound had a docking score of −8.637 kcal/mol and was bound with SARS-CoV-2 Nsp12. The respective compound interacts with Thr701, Gln789, and Tyr732 residues. In Thr701, (H…OH) hydrogen interacted with the oxygen at a distance of 1.86 Ǻ. In Gln789, (H…OH) hydrogen interacted with the oxygen group at a distance of 1.88 Ǻ. In Tyr732, (H…OH) hydrogen interacted with the oxygen group at a distance of 2.16 Ǻ. The residues interactions play a major role in SARS-CoV-2 protein antagonist activity.

### 3.4. Virtual Screening Study of SARS-CoV-2 Structural and Nonstructural Proteins with Kabasura Kudineer Compounds

A huge set of Kabasura Kudineer compounds were docked with structural and nonstructural SARS-CoV-2 proteins. As a result, when compared to other compounds, the Kabasura Kudineer compounds, namely, 250395, 129677029, 44259583, 44259584, and 88583189, had an excellent scoring function with SARS-CoV-2 protein. The 44259583 compound has a high binding score when compared to the other five compounds. The binding score of compound 44259583 was –13.759, kcal/mol with SARS-CoV-2 Nsp12, as shown in Table 2.

### 3.5. Binding Mode Analysis of the Kabasura Kudineer Compound

The binding modes of the best compounds were analyzed by the Glide XP module. The binding mode analysis of the best five compounds image is given in Figure 2.

#### 3.5.1. Binding Mode Analysis of the Compound 250395

The docking score of 250395 compounds was −11.094 kcal/mol and was bound with SARS-CoV-2 spike protein. The respective compound interacts with Arg355, Thr430, and Asp428 residues. In Arg355, (H…OH) hydrogen interacted with the oxygen group at a distance of 2.70 Ǻ. In Thr430, (H…OH) hydrogen interacted with the oxygen group at a distance of 1.93 Ǻ. In Asp428, (H…OH) hydrogen interacted with the oxygen group, at a distance of 1.91 Ǻ, and in the same residues, (H…OH) hydrogen interacted with the oxygen group at a distance of 1.85 Ǻ. The residues interactions play a major role in SARS-CoV-2 protein antagonist activity.

RETRACTED

#### 3.5.2. Binding Mode Analysis of the Compound 129677029

The docking score of 129677029 compounds was −7.273 kcal/mol and was bound with SARS-CoV-2 membrane protein. The respective compound interacts with Phe112, Ser111, Ser108, and Phe103 residues. In Phe112, (H…OH) hydrogen interacted with the oxygen group at a distance of 1.90 Ǻ. In Ser111, (H…OH) hydrogen interacted with the oxygen group, which distance is 2.37 Ǻ. In Ser108, (H…OH) hydrogen interacted with the oxygen group at a distance of 1.80 Ǻ. In Phe103, (H…OH) hydrogen interacted with the oxygen group at a distance of 1.98 Ǻ. The residues interactions play a major role in SARS-CoV-2 protein antagonist activity.

#### 3.5.3. Binding Mode Analysis of the Compound 44259583

The docking score of 44259583 compounds was −11.688 kcal/mol and was bound with SARS-CoV-2 Nsp14. The respective compound interacts with Lys93, Lys95, Asn40, Thr5, Ala71, and Cys77 residues. In Lys93, (H…OH) hydrogen interacted with the oxygen group of 44259583 compound at a distance of 2.36 Ǻ. In Lys95, (H…OH) hydrogen interacted with the oxygen at a distance of 1.99 Ǻ. In Asn40, (H…OH) hydrogen interacted with the oxygen group at a distance of 2.07 Ǻ, and the same residues of (H…OH) hydrogen interacted with the oxygen group at a distance of 1.89 Ǻ. In Thr5, (H…OH) hydrogen interacted with the oxygen group at a distance of 1.78 Ǻ. In Ala71, (H…OH) hydrogen interacted with the oxygen group at a distance of 2.62 Ǻ. In Cys77, (H…OH) hydrogen interacted with the oxygen group at a distance of 2.13 Ǻ. The residues interactions play a major role in SARS-CoV-2 protein antagonist activity.

#### 3.5.4. Binding Mode Analysis of the Compound 44259584

The docking score of 44259584 compounds was −11.450 kcal/mol and was bound with SARS-CoV-2 Nsp14. The respective compound interacts with Thr5, His80, Cys77, Lys93, and Asn40 residues. In Thr5, (H…OH) hydrogen interacted with the oxygen group at a distance of 1.73 Ǻ, and in the same residues, (H…OH) hydrogen residues interacted with the oxygen group at a distance of 1.82 Ǻ. In His80, (H…OH) hydrogen interacted with the oxygen at a distance of 1.77 Ǻ. In Cys77, (H…OH) hydrogen interacted with the oxygen group at a distance of 2.30 Ǻ. In Lys93, (H…OH) hydrogen interacted with the oxygen group at a distance of 1.73 Ǻ. In Asn40, (H…OH) hydrogen interacted with the oxygen group at a distance of 2.01 Ǻ, and in the same residues, (H…OH) hydrogen interacted with the oxygen group at a distance of 2.03 Ǻ. The residues interactions play a major role in SARS-CoV-2 protein antagonist activity.

RETRACTED

#### 3.5.5. Binding Mode Analysis of the Compound 44259583

The docking score of 44259583 compounds was −10.850 kcal/mol and was bound with SARS-CoV-2 Nsp13. The respective compound interacts with Asp534, Ser535, Gln537, and Asp383 residues. In Asp534, (H…OH) hydrogen interacted with the oxygen group at a distance of 1.91 Ǻ. In Gln537, (H…OH) hydrogen interacted with the oxygen group at a distance of 2.26 Ǻ, and in the same residues, (H…OH) hydrogen interacted with the oxygen group at a distance of 1.74 Ǻ. In Ser535, (H…OH) hydrogen interacted with the oxygen group at a distance of 1.67 Ǻ. In Asp383, (H…OH) hydrogen interacted with the oxygen group at a distance of 1.96 Ǻ, and the same residues of (H…OH) hydrogen interacted with the oxygen group, which distance is of 1.95 Ǻ. The residues interactions play a major role in SARS-CoV-2 protein antagonist activity.

#### 3.5.6. Binding Mode Analysis of the Compound 44259584

The docking score of 44259584 compound was −13.337 kcal/mol and was bound with SARS-CoV-2 main protease. The respective compound interacts with Glu166, Leu141, Asn142, His41, and Thr26 residues. In Glu166, the residues were formed by three hydrogen bond interactions with 44259584 compounds. In Glu166, (H…OH) hydrogen interacted with the oxygen at a distance of 1.98 Ǻ; (H…OH) hydrogen interacted with the oxygen group at a distance of 1.84 Ǻ; and (H…OH) hydrogen interacted with the oxygen group at a distance of 2.63 Ǻ. In Leu141, (H…OH) hydrogen interacted with the oxygen group at a distance of 2.07 Ǻ. In His411, pi-pi stacking was formed. In Asn142, (H…OH) hydrogen interacted with the oxygen group at a distance of 1.80Ǻ. In Thr26, (H…OH) hydrogen interacted with the oxygen group at a distance of 2.12 Ǻ, and in the same residues, (H…OH) hydrogen residues interacted with the oxygen group at a distance of 2.19 Ǻ. The residues interactions play a major role in SARS-CoV-2 protein antagonist activity.

#### 3.5.7. Binding Mode Analysis of the Compound 44259583

The docking score of 44259583 compound was −13.759 kcal/mol and was bound with SARS-CoV-2 Nsp15. The respective compound interacts with Tyr279, Ser274, Asp273, Leu201, Asp268, Gly165, Lys90, and Tyr89 residues. In Tyr279, (H…OH) hydrogen interacted with the oxygen group of compound 44259583 at a distance of 2.32 Ǻ. In Ser274, (H…OH) hydrogen interacted with the oxygen at a distance of 1.89 Ǻ, and in the same residues, (H…OH) hydrogen interacted with the oxygen group at a distance of 2.61 Ǻ. In Asp273, (H…OH) hydrogen interacted with the oxygen group at a distance of 1.79 Ǻ. In Leu201, (H…OH) hydrogen interacted with the oxygen group at a distance of 2.02 Ǻ. In Asp268, (H…OH) hydrogen interacted with the oxygen group at a distance of 2.65 Ǻ, and in the same residues, (H…OH) hydrogen interacted with the oxygen group at a distance of 2.05 Ǻ. In Gly165, (H…OH) hydrogen interacted with the oxygen group at a distance of 1.91 Ǻ, and in the same residues, (H…OH) hydrogen interacted with the oxygen group at a distance of 1.92 Ǻ. In Lys90, residues had pi-pi interactions; this pi-pi interaction was strong for stable binding of the compound in the active site of SARS-CoV-2. In Tyr89, (H…OH) hydrogen interacted with the oxygen group at a distance of 2.21 Ǻ. The residues interactions play a major role in SARS-CoV-2 protein antagonist activity.

RETRACTED

#### 3.5.8. Binding Mode Analysis of the Compound 44259584

The docking score of 44259584 compounds was −13.791 kcal/mol and was bound with SARS-CoV-2 Nsp15. The respective compound interacts with Tyr89, Lys90, Asp268, Tyr279, and Ser198 residues. In Tyr89, (H…OH) hydrogen interacted with the oxygen group of compound 3802778 at a distance of 1.60 Ǻ, and in the same residues, (H…OH) hydrogen interacted with the oxygen group at a distance of 1.71 Ǻ. In Lys90, (H…OH) hydrogen interacted with the oxygen at a distance of 1.76 Ǻ. In Asp268, (H…OH) hydrogen interacted with the oxygen group at a distance of 1.76 Ǻ. In Tyr279, (H…OH) hydrogen interacted with the oxygen group at a distance of 2.13 Ǻ, and In Ser198, (H…OH) hydrogen interacted with the oxygen group at a distance of 1.91 Ǻ. The residues interactions play a major role in SARS-CoV-2 protein antagonist activity.

#### 3.5.9. Binding Mode Analysis of the Compound 88583189

The 88583189 compound is having a docking score of −8.290 kcal/mol and binds with SARS-CoV-2 Nsp12. The respective compound interacts with Arg132, Gln789, and Asn705 residues. In Arg132, (H…OH) hydrogen interacted with the oxygen at a distance of 2.58 Ǻ. In Gln789, (H…OH) hydrogen interacted with the oxygen group at a distance of 2.06 Ǻ. In Asn705, (H…OH) hydrogen interacted with the oxygen group at a distance of 1.86 Ǻ. The residues interactions play a major role in SARS-CoV-2 protein antagonist activity.

### 3.6. Density Function Theory (DFT) Calculations of Kabasura Kudineer and Homeopathy Compounds

The top hit compounds were subjected for DFT calculation done by the Jaguar version 7.8 (Schrödinger, LLC, New York, NY, 2018-4). The HOMO and LUMO values were calculated for homeopathy compounds, and the values ranged from −0.217 to −0.237 and −0.006 to −0.0706, as shown in Table 3 and Figure 3. HOMO and LUMO values represent electron donation and acceptance. In compounds 38021778 and 32036, the HOMO and LUMO regions are in the aromatic ring region. In compound 5315852, the HOMO regions are located in the ring moiety, and LUMO regions are present in the functional groups. In compounds 14590080 and 7402975, HOMO and LUMO regions are situated in the functional group's moiety. In compounds 250395 and129677029, HOMO and LUMO energy were located on the aromatic regions. The 44525958, 44259584, and 88583189 compounds have the electron transfer in the functional group's moiety. Based on the results, our compounds have high HOMO regions that acted as nucleophile effect to the target, and electrophilic effect is high in the LUMO region. The results of HOMO and LUMO findings showed that the ligands have a higher electron donor and acceptor activity. The HOMO and LUMO are well correlated to the docking outcomes. The electron donor and acceptor range of ligands was determined using the HOMO and LUMO values. The Kabasura Kudinner compounds' HOMO and LUMO values ranged from −0.216 to −0.234 and −0.0355 to −0.067, which are shown in Table 4 and Figure 4. The molecule's chemical activity affects the energy gap of HOMO and LUMO. The decreased energy gap shows the intramolecular charge transfer and kinetic stability. Here, all the molecules have lower HOMO-LUMO gap energy that explicitly, all the compounds are chemically reactive and served as an activity with the target.

RETRACTED

#### 3.6.1. Molecular Electrostatic Potential (MESP) and Solvation Energy Calculation

The stereoelectronic matching of receptor and ligand is critical for classifying protein-ligand interactions at the molecular level. The surface characteristics of lead compounds were sorted out using the 3D-MESP parameters and others, which were beneficial in mentioning the ligand pharmacophore attribute and their surface, which play a significant part in binding. The most negative potential regions indicate the attraction of protons and positive indicates the repulsion of a proton within the molecule. The calculated MESP values show that all the compounds have good proton transferability. Especially, the best five homeopathy compounds have more proton attraction ability. Meanwhile, the Kabasura Kudineer compounds have more proton repulsion within the target. The functional groups of all the compounds have the most positive potential that shares the electron to the target. The aromatic ring region has a negative potential that allows for electron acceptance. Hence, the MESP analysis shows the region for electrophilic and nucleophilic attack, and this region makes hydrogen bonds with the target. The solvation energy is crucial for molecular recognition, macromolecular interaction, aqueous stability, and sustainability. The drug interaction differs from the solvent and changes the molecule to strong interaction with the target. Here, all the molecules have good solvation energy, which explicit the compounds that can interact with SARS-CoV2 proteins and make electron transferring with the target [30]. The best five Kabasura Kudineer and homeopathy compounds, stereoelectronic property of MESP, and others such as HOMO, LUMO, and salvation energy were identified and are shown in Tables 3 and 4, and MESP Iso-surface is shown in Figures 5 and 6.

RETRACTED

As a result, we determine the ligand's solvation energy, which was critical in computing compound aqueous solubility. The top hit Kabasura Kudineer compound solvation energies vary from −0.11 to −121.60 as shown in Table 2, while the best hit homeopathy compounds solvation energies ranged from −13.16 to −71.41 in Tables 3 and 4. The salvation energy values were more negative in range, which represents that the compounds were having more aqueous solubility.

### 3.7. ADME/T Property Analysis

The Schrödinger QikProp module proved helpful in categorizing drug-likeness (Lipinski's rule of five) and ADME (absorption, distribution, metabolism, and excretion) characteristics. The discovered Kabasura Kudinner and homeopathic compounds were found to have physically significant characteristics as well as pharmaceutically relevant capabilities (Merz, Ringe, and Reynolds, 2010). The drug-likeness descriptors such as molecular weight, QPPCaco, QPLog HERG, LogP Po/w (octanol/water), LogP MDCK, and percentage of human oral absorption based on Lipinski's rule of five point out that the compounds are at an acceptable range.

#### 3.7.1. ADME Properties of the Homeopathy Compounds

The homeopathic component QPlogPo/w (partition coefficient) was ranging from −0.97 to 1.02, which was used to estimate the medication absorption and distribution across the body, and QPPCaco value ranging from 0.29 to 58.42 governs the cell permeability factor and also affects a drug's metabolic activity. The Qplog HERG varies from −3.35 to −5.62, and the QPPMDCK ranges from 0.09 to 22.97. The human oral absorption (HOA) of three compounds varied from 13.8 to 54.48% as indicated in Table 5.

#### 3.7.2. ADME Properties of the Kabasura Kudineer Compounds

The Kabasura Kudineer component QPlogPo/w (partition coefficient) was ranging from −1.42 to 0.06 and was used to estimate the medication absorption and distribution across the body, and QPPCaco value ranging from −0.05 to 1127.6 governs the cell permeability factor that affects a drug's metabolic activity. The Qplog HERG varies from −3.69 to −6.16, and the QPPMDCK value ranges from 0.01 to 563.32. The human oral absorption (HOA) of three compounds varies from 56.43 to 89.88%, as indicated in Table 6. Overall, the pharmacokinetic activities of Kabasura Kudineer and homeopathic components were drug-like and suitable for human usage. These compounds were taken to precede a clinical trial to examine good results.

RETRACTED

### 3.8. Molecular Dynamics Simulation

For molecular dynamics simulations, protein-ligand complexes were considered. In complex dynamics, computational methods were more valuable for evaluating protein flexibility and releasing the dynamics model. Furthermore, we identified that the methods were quite stable, and the simulations were in the acceptable range for further process.

#### 3.8.1. Root-Mean-Square Deviation (RMSD) Analysis

The magnitude of confirmation drift of the protein was assessed using the root-mean-square deviation (RMSD) of backbone atoms as a function of time in the array concerning the starting structure (Figure 7). The RMSD plots of Nsp14 complexes have maintained stability within 4 to 6 Å throughout the simulation period. In Nsp13 complexes, the 44259584 and 74029795 compounds have maintained stability in the range of 2 to 3.5 Å, but the 74029745 complex has slight fluctuation in the 40 to 80 Å and attains its stability in below 5.0 Å in 100 ns time interval. The main protease complexes have maintained stability throughout the simulation time within 1.5 to 2.5 Å time intervals. Nsp15 with 44259584 and 44259583 complexes has maintained stability within 1.5 to 2.5 Å, but less fluctuation was observed in 70 to 85 ns time interval for 3802778 and Nsp15 complex, and then it was stable in 100 ns interval (3.0 Å). The Nsp12 complexes have maintained stable conformation within 2.0 Å to 3.0 Å throughout the simulation period. In spike protein, the small deviation was observed in 3802778 in 50 to 60 ns time interval, and it maintains stable form in 80 to 100 ns time interval, as well as the compound 250395 maintains the stable conformation in the range of 1.25 to 2.0 Å. The membrane protein complex 320361 attains stability of 1.5 to 2.0 Å throughout the simulation period. But slight fluctuation was observed in 320361 compound in the range of 25 to 40 ns time interval, and it attains stability in 2.0 Å. Overall, the RMSD plot depicts all the complexes have not fluctuated significantly. All complexes have attained the deviation in the range of 2.0 to 5.0 Å, especially some of the complexes that have 1.5 to 2.5 Å deviation, which clearly shows that the selected compound has well bound to the respective proteins and maintains the stable conformation throughout the simulation time interval.

RETRACTED

#### 3.8.2. Root-Mean-Square Fluctuation (RMSF) Analysis

The RMSF value indicates how ligand binding might affect protein conformation followed by binding conformation. The RMSF value of inflexible structures such as helix and sheets was low, but the RMSF value of slack structures such as sheets and turns was high. The residue flexibility in the SARS-CoV-2 structural and nonstructural proteins was determined by the molecular dynamics simulations shown in Figure 8. The RMSF plot of the Nsp14 complex revealed that 80–100 residues have high fluctuation, and the remaining residues have less fluctuation within 2.5 Å. The residues from 50 to 100 have higher fluctuation in Nsp13 complex, and slight fluctuation was observed in 400–500 residues that occur in the nonactive site region of Nsp13 and the active site region having less fluctuation. The main protease complexes depict their maintaining stability within a range of 0.5 to 2.0 Å throughout the simulation period. In Nsp15 protein complex, 170–180 residues have slight fluctuations were noted, and their remaining residues had below 2.4 Å in a simulation period. In 320361 with Nsp12 complex, the residues between 600 and 620 show higher fluctuation and the 8858189 with Nsp12 complex shows fluctuation in the 140–155 and 180–185 residue regions. These fluctuations are in the loop region and are not affected by the complex stability. Membrane protein complex analysis revealed that not much fluctuation was noted, and the fluctuation ranges from 0.5 to 2.0 Å. Overall, the RMSF analysis revealed that the active site residues have less function in the range of 0.5 to 2.5 Å, and the nonactive site regions have higher fluctuation. All the complexes have maintained stable conformation throughout the simulation period.

#### 3.8.3. Hydrogen Bond Analysis

During the simulation period, the time dependency of hydrogen bonds between receptor and drug-like molecules was studied in order to estimate the drug molecule binding rate at the active site of SARS-CoV-2 structural and nonstructural proteins (Figure 9). According to the findings, the discovered intermolecular hydrogen bonding was linked to the biological actions of its best inhibitory drugs. The Kabasura Kudineer and homeopathy compounds have stable hydrogen bonding interactions for the period of the simulation time, and this gave an intimation on its appeal towards the protein-ligand complexes.

## 4. Conclusion

SARS-CoV-2 is a sheathed, constructive sense, single-stranded RNA virus-like SARS (severe acute respiratory syndrome). This virus contains many targets of structural proteins such as membrane protein, spike protein, and nonstructural proteins including main protease, Nsp12 (RNA-dependent RNA polymerase), Nsp13 (helicase), Nsp14 (exonuclease), and Nsp15 (uridylate); these are the most important targets of COVID-19. In this study, we tried all the possibilities to include SARS-CoV-2 structural and nonstructural proteins as targets through multitargeted way viral replications, and hence, further spread can be controlled. The Kabasura Kudinner is multiherbal mixture; most of the compounds are water-soluble; each compound act on different site viral targets; and also, it boosts up the immunity of the individuals. The virtual screening workflow was carried out for SARS-CoV-2 structural and nonstructural proteins. Overall, 14,682 Kabasura Kudinner and 3,112 homeopathy compounds were docked with targeted proteins; 192 Kabasura Kudinner compounds and 192 homeopathy compounds were screened against SARS-CoV-2 structural and nonstructural protein. As a result, five compounds of Kabasura Kudineer, namely, 250395, 129677029, 44259583, 44259584, and 88583189 (Kabasura Kudineer), and five homeopathy compounds such as 3802778, 320361, 5315832, 14590080, and 74029795 were chosen since they had a good binding score and binding energy compared to other compounds. While the DFT result revealed a result of the top five compounds with high electron donor and acceptor regions. These regions in the compounds make hydrogen bond interactions with SARS-CoV-2 structural and nonstructural protein. HOMO-LUMO gap also exposed that these compounds are highly reactive in nature. The molecular dynamics simulation exposed that the compounds precisely fit into the protein and were more stable in nature. Overall, the machinery actions of the phytocompounds (250395, 129677029, 44259583, 44259584, and 88583189 (Kabasura Kudineer) and the 3802778, 320361, 5315832, 14590080, and 74029795 (homeopathy)) present in the Kabasura Kudineer and homeopathy formulations were binding with many amino acids at various sites of the SARS-CoV-2 structural and nonstructural proteins. Therefore, these compounds have best inhibitory function against SARS-CoV-2 structural and nonstructural proteins. This computational study helps understand the inhibition mechanism of Kabasura Kudineer and homeopathy compounds against SARS-CoV-2 proteins. Our future work will focus on applying these compounds in omicron variants and confirming their binding stability and conformational changes, as well as examining their inhibitory effects *in vitro* and *in vivo* against SARS-CoV-2.

RETRACTED

## Figures and Tables

**Figure 1:** The 2D interaction binding mode of homeopathy compounds with SARS-CoV-2 proteins. The pink color arrow represents the hydrogen bond interaction.

**Figure 2:** The 2-D interaction binding mode of Kabasura Kudineer compounds with SARS-CoV-2 proteins. The pink color arrow represents the hydrogen bond interactions, and the red color represents the Pi-cation interaction.

**Figure 3:** HOMO and LUMO mapping of 3802778 (a, b), 32036 (c, d), 5315832 (e, f), 14590080 (g, h), and 74029795 (i, j) homeopathy compounds. Blue and red color regions represent positive and negative potential, respectively.

**Figure 4:** HOMO and LUMO mapping of 250395 (a, b), 129677029 (c, d), 44259583 (e, f), 4425984 (g, h), and 88583189 (i, j) Kabasura Kudineer compounds. Blue and red color regions represent positive and negative potential, respectively.

**Figure 5:** MESP mapping of 3802778 (a), 32036 (b), 5315832 (c), 14590080 (d), and 74029795 (e) homeopathy compounds. The most negative electrostatic potential was colored deepest red, and the most positive electrostatic potential was colored deepest blue. The intermediate yellow, orange, and green shades indicate the ranges of reactivity.

**Figure 6:** MESP mapping of 250395 (a), 129677029 (b), 44259583 (c), 4425984 (d), and 88583189 (e) Kabasura Kudineer compounds. The most negative electrostatic potential was colored deepest red, and the most positive electrostatic potential was colored deepest blue. The intermediate yellow, orange, and green shades indicate the ranges of reactivity.

**Figure 7:** RMSD plot of SARS-CoV-2 proteins and screened compound complexes. Nsp14 (a), Nsp13 (b), main protease (c), Nsp15(d), Nsp12 (e), spike (f), and membrane protein (g).

**Figure 8:** RMSF plots of SARS-CoV-2 proteins and screened compound complexes. Nsp14 (a), Nsp13 (b), main protease (c), Nsp15 (d), Nsp12 (e), spike (f), and membrane protein (g).

**Figure 9:** Histogram of hydrogen bond contact of top hit Kabasura Kudineer and homeopathy compounds with SARS-CoV-2 proteins. Hydrogen bonds are represented by green color, hydrophobic by purple, ionic bonds by pink, and water bridges by blue.

**Table 1:** Glide score and glide energy of homeopathy compounds with SARS-CoV-2 structural and nonstructural proteins.

Structural protein			
Plant name	Compound ID	Glide score (kcal/mol)	Glide energy (kcal/mol)
Spike protein (PDB: ID 7BZ5)			
Arnica flowers	3802778	−7.929	−47.657
Membrane protein			
Arnica flowers	320361	−5.636	−37.056

Nonstructural protein			
Plant name	Compound ID	GLIDE score (kcal/mol)	Glide energy (kcal/mol)
Nsp14 (PDB: ID 5C8S)			
Arnica flowers	3802778	−9.583	−57.967
Arnica flowers	5315832	−7.672	−40.340
Nsp13 (PDB: ID 5WWP)			
Pulsatila	14590080	−13.631	−75.093
Pulsatila	74029795	−11.957	−71.614
Main protease (PDB: ID 6LU7)1			
Pulsatila	74029795	−10.970	−61.272
Nsp15 (PDB: ID 6X4I)			
Arnica flowers	3802778	−10.902	−59.517
Nsp12 (PDB: ID 6XQB)			
Arnica flowers	320361	−8.637	−37.064

RETRACTED

**Table 2:** Glide score and glide energy of homeopathy compounds with SARS-CoV-2 structural and nonstructural proteins.

Kabasura Kudineer compounds			
Structural protein			
Plant name	Compound ID	Glide score (kcal/mol)	Glide energy (kcal/mol)
Spike protein (PDB: ID 7BZ5)			
*Terminalia chebula*	250395	−11.094	−47.778
Membrane protein			
*Syzygium aromaticum*	129677029	−7.273	−26.721

Kabasura Kudineer compounds			
Nonstructural protein			
Plant name	Compound ID	Glide score (kcal/mol)	Glide energy (kcal/mol)
Nsp14 (PDB: ID 5C8S)			
*Syzygium aromaticum*	44259583	−11.688	−65.163
*Syzygium aromaticum*	44259584	−11.450	−57.323
Nsp13 (PDB: ID 5WWP)			
*Syzygium aromaticum*	44259583	−10.850	−74.079

Main protease (PDB: ID 6LU7)			
*Syzygium aromaticum*	44259584	−13.337	−81.395
Nsp15 (PDB: ID 6X4I)			
*Syzygium aromaticum*	44259583	−13.759	−77.222
*Syzygium aromaticum*	44259584	−13.791	−75.686
Nsp12 (PDB: ID 6XQB)			
*Coleus amboinicus*	88583189	−8.290	−45.199

**Table 3:** HOMO, LUMO, solvation energy, and MESP of top hit homeopathy compounds.

Compound ID	HOMO (eV)	LUMO (eV)	Solvation energy (kcal/mol)	MESP (kcal/mol)	
				Most negative potential	Most positive potential
7402935	−0.233	−0.006	−0.11	−66.59	105.98
320361	−0.234	−0.067	−29.27	−54.43	65.38
3802778	−0.217	−0.0706	−121.60	−187.23	47.84
5315832	−0.218	−0.069	−107.41	−183.69	56.04
14590080	−0.237	−0.0147	−78.15	−60.35	66.97

**Table 4:** HOMO, LUMO, solvation energy, and MESP of top hit Kabasura Kudineer compounds.

Compound ID	HOMO (eV)	LUMO (eV)	Solvation energy (kcal/mol)	MESP (kcal/mol)	
				Most negative potential	Most positive potential
44259583	−0.219	−0.0644	−71.41	−69.12	67.30
44259584	−0.216	−0.0615	−68.78	−73.24	69.46
88583189	−0.257	−0.0355	−28.64	−68.39	77.91
250395	−0.221	−0.054	−66.87	−57.96	63.27
129677029	−0.226	−0.046	−13.16	−36.80	46.73

**Table 5:** ADME properties of the homeopathy compounds.

Compound ID	Molecular weight (g/mol)	Qplog po/w	Qplog HERG	QppCaco	QppMDCK	Rule of five	HOA	Percentage of HOA
3802778	516.45	1.02	−4.99	0.36	0.12	3	1	0
5315832	354.3	−0.34	−3.35	1.27	0.46	1	1	13.8
14590080	1,221.3	−3.49	−5.62	0.57	0.15	3	1	0
7402935	1,075.2	−2.17	−3.76	5.52	1.79	3	1	0
320361	324.3	−1.01	−4.82	50.27	19.52	0	2	54.48

**Table 6:** ADME properties of the Kabasura Kudineer compounds.

Compound ID	Molecular weight (g/mol)	Qplog po/w	Qplog HERG	QppCaco	QppMDCK	Rule of five	HOA	Percentage of HOA
250395	636.47	−2.83	−5.34	−0.05	0.01	3	1	0
129677029	198.21	−1.42	−3.69	1127.6	563.32	0	3	89.88
88583189	302.36	0.06	−4.49	42.47	16.27	0	2	56.43
44259583	802.69	−4.61	−5.81	0.78	0.04	3	1	0
44259584	812.73	−2.06	−6.16	2.08	0.62	2	1	0

RETRACTED

## Data Availability

The data used to support the findings of this study are included in the article.

## Supplementary Materials

Supplementary Materials Figures S1-S2: Kabasura Kudineer and homeopathy ingredients. Table S1-S2: benefits of Kabasura Kudineer and homeopathy ingredients.
